The article "Construction and Simulation of Biomechanical Model of Human Hip Joint Muscle-Tendon Assisted by Elastic External Tendon by Hill Muscle Model" was published in 2022. Journal: Comput Intell Neurosci.

# Construction and Simulation of Biomechanical Model of Human Hip Joint Muscle-Tendon Assisted by Elastic External Tendon by Hill Muscle Model

**DOI:** 10.1155/2022/1987345

**Published:** 2022-08-02

**Authors:** Xi Luo, Guofeng Cai, Kun Ma, Aiqi Cai

**Affiliations:** ^1^Faculty of Civil Engineering and Mechanics, Kunming University of Science and Technology, Kunming 650500, Yunnan, China; ^2^Department of Sports Medicine, First Affiliated Hospital of Kunming Medical University, Kunming 650032, Yunnan, China; ^3^Department of Medical Genetics, First People's Hospital of Yunnan Province (The Affiliated Hospital of Kunming University of Science and Technology), Kunming 650032, Yunnan, China

## Abstract

Based on the Hill muscle model (HMM), a biomechanical model of human hip muscle tendon assisted by elastic external tendon (EET) was preliminarily established to investigate and analyze the biomechanical transition between the hip joint (HJ) and related muscle tendons. Using the HMM, the optimal muscle fiber length and muscle force scaling variables were introduced by means of constrained optimization problems and were optimized. The optimized HMM was constructed with human parameters of 170 cm and 70 kg. The biomechanical model simulation test of the hip muscle tendon was performed in the automatic dynamic analysis of mechanical systems (ADAMS) software to analyze and optimize the changes in the root mean square error (RMSE), biological moment, muscle moment distribution coefficient (MDC), muscle moment, muscle force, muscle power, and mechanical work of the activation curves of the hip major muscle, iliopsoas muscle, rectus femoris muscle, and hamstring muscle under analyzing the optimized HMM and under different EET auxiliary stiffnesses from the joint moment level, joint level, and muscle level, respectively. It was found that the trends of the output joint moment of the optimized HMM and the biological moment of the human HJ were basically the same, *r*^2^ = 0.883 and RMSE = 0.18 Nm/kg, and the average metabolizable energy consumption of the HJ was (243.77 ± 1.59) J. In the range of 35%∼65% of gait cycle (GC), the auxiliary moment showed a significant downward trend with the increase of EET stiffness, when the EET stiffness of the human body was less than 200 Nm/rad, the biological moment of the human HJ gradually decreased with the increase of EET stiffness, and the MDC of the iliopsoas and hamstring muscles gradually decreased; when the EET stiffness was greater than 200 Nm/rad, the increase of the total moment of the extensor muscles significantly increased, the MDC of the gluteus maximus and rectus muscles gradually increased, and the gluteus maximus and hamstring muscle moments and muscle forces gradually increased; the results show that the optimized muscle model based on Hill can reflect the law of human movement and complete the simulation test of HJ movements, which provides a new idea for the analysis of energy migration in the musculoskeletal system of the lower limb.

The article "Construction and Simulation of Biomechanical Model of Human Hip Joint Muscle-Tendon Assisted by Elastic External Tendon by Hill Muscle Model" was published in 2022. Journal: Comput Intell Neurosci.

## 1. Introduction

All joints and muscles of the human lower limb are involved in the process of natural walking, and the dynamics between each joint and muscle are in the process of change during a complete change cycle, and the structural characteristics of the body's joints and their corresponding movement characteristics are the basis of exoskeleton activity [1]. Elastic elements play an important role in the activity of the musculoskeletal system of the lower extremities, while they can have a significant effect on limb metabolic energy consumption (EC) [2]. The hip joint (HJ) is the largest positive work joint in the human lower limb, with stability and a large range of motion [3], and plays an important role in human walking and maintaining body balance [4]. The HJ is mainly composed of two parts: pelvis and femur, which are connected through femoral head and acetabulum. Approximately 21 muscles participated in the movement during the movement of the HJ. The extensor and flexor muscle groups of the HJ cooperate with each other to jointly control the activities of various joints of the human lower limb, and elastic tissues such as ligaments in the human. HJ can assist the muscle tissue to support the movement of the human body [5]. Previous findings have pointed out that during walking, when the body's auxiliary joints show positive work, they can significantly reduce body EC [6]. In addition, it has been pointed out that even if the body's auxiliary joints show negative work, the body EC can be similarly reduced by providing damping assistance [7]. Elastic external tendon (EET) tissue has significant characteristics of storing energy and releasing energy, and body energy can be effectively reduced by sharing part of the muscle force during walking or exercise in the lower limbs [8].

In recent years, HJ has received much attention in orthopedic clinical and biomechanical research. The research on the transport biomechanical model of human HJ belongs to the research category of sports biomechanics, which has a wide range of research scope, mainly including biology and metrology, the establishment of biomechanical model, and the computer simulation of biological movement mechanism. Among them, the research of the human body is an important direction in sports biomechanics, which is mainly achieved by modeling. At present, biomechanical models of the HJ have been widely used in biology and biological motion machine simulation [9]. The human joint model is based on motion mechanics, and the research methods of motion biomechanics mainly include the application of multi-body theory to establish kinetic model and human simulation research. Muscle model is an important part of human biomechanical model to explore the musculoskeletal system, and the commonly used muscle motor system models are Hill theoretical, Huxley, and rheological models [10]. Based on the relationship between thigh muscle contraction and heat production in frogs, British physiologist Hill proposed the theory of Hill muscle contraction, which is the theoretical basis for the study of skeletal muscle dynamics and has been widely used in lower limb modeling [11]. The researchers applied Hill theory to skeletal muscle, tendon, and human movement control and established a Hill muscle model (HMM) [12]. The human muscle system is complex, and the biomechanics of the muscle system as well as the analysis of interactions between muscles are difficult. The traditional HMM lacks the measurement of physiological parameters such as the degree of muscle activation and is severely limited during use [13]. Although the optimization algorithm based on Hill theory can evaluate the muscle force in the movement of the musculoskeletal system.Its accuracy is limited, and forward dynamics calculation cannot be performed [14]. At present, scholars have established muscle mechanical models, but most of these models are test-based and mostly physiological models rather than biomechanical models [15]. Passive bone simulation based on energy conversion and migration in the human musculoskeletal system and assisted by EET is still a challenging problem in passive exoskeleton design. Therefore, it is of great significance to establish a biomechanical model of the HJ with relatively few parameters and clear mechanical meaning for orthopedic clinical and biomechanical studies.

The article "Construction and Simulation of Biomechanical Model of Human Hip Joint Muscle-Tendon Assisted by Elastic External Tendon by Hill Muscle Model" was published in 2022. Journal: Comput Intell Neurosci.

Therefore, based on the HMM, the biomechanical model of human hip muscle tendon assisted by EET was preliminarily established by optimizing it, and the simulation experiment was performed based on the model to investigate the biomechanical transition among the HJ and related muscle tendons, providing a new idea for the analysis of hip biomechanics and energy migration of the lower limb musculoskeletal system.

## 2. Materials and Methods

### 2.1. HMM

The HMM was used to model a single muscle, which was often expressed as muscle-tendon unit (MTU) and was mainly composed of three parts: contractile element (CE), parallel element (PEE), and series element (SEE) [16]. CE refers to the active force generated by the action within the muscle; PEE refers to the passive tension generated within the muscle; SEE refers to the elastic tendon tissue that connects the muscle to the bone. The calculation method of the passive tendon force of SEE in the HMM can be expressed as follows:

(1) $$\begin{array}{c} F_{T}=F_{\text{MUT}}\cos\;\alpha =\left(F_{CE}+F_{\text{PEE}}\right)\cos\;\alpha , \end{array}$$

*F*_*CE*_ indicates the active force generated by *CE* when subjected to nerve stimulation; *F*_PEE_ indicates the passive tension; *α* is the pinna angle; *F*_MUT_ is the muscle force of MTU; *F*_*T*_ indicates the passive tendon force of *SEE*.

The MT length is calculated as follows:

(2) $$\begin{array}{c} L_{MT}=L_{\text{MUT}}\cos\;\alpha +L_{T}, \end{array}$$

*L*_MUT_ indicates the actual length of the muscle fiber; *L*_*T*_ indicates the length of *SEE*; *L*_*MT*_ indicates the MT; *α* is the pinna angle.

When *α*=0, the tendon force and tendon length in the HMM can be expressed as follows:

(3) $$\begin{array}{c} F_{T}=F_{\text{MUT}}=F_{CE}+F_{\text{PEE}}\text{,} \end{array}$$

(4) $$\begin{array}{c} L_{MT}=L_{\text{MUT}}+L_{T}. \end{array}$$

Human movement is based on the mechanical properties of skeletal muscle [17]. The generation of *F*_*CE*_ follows the myofilament sliding theory. The generation of *F*_*CE*_ is related to the actual length *L*_MUT_, contraction speed *V*_MUT_, and activation degree *α* of muscle fibers.

(5) $$\begin{array}{c} F_{CE}=F_{\max}\cdot \tilde{F_{CE}}=F_{\max}\cdot \alpha \tilde{f_{CE}}\left(\tilde{L_{\text{MUT}}}\right)\cdot \tilde{f_{CE}}\left(\tilde{V_{\text{MUT}}}\right), \end{array}$$

*F*_max_ is the maximum muscle force that can be generated during muscle isometric contraction, and $\tilde{F_{CE}}$ is the normalized active muscle force after the maximum isometric *F*_max_ normalization of *F*_*CE*_. $\tilde{L_{\text{MUT}}}$ is the standardized muscle fiber length after *L*_*MUT*_ normalized by the optimal muscle fiber length *L*_0_^*m*^, and $\tilde{V_{\text{MUT}}}$ is the standardized muscle fiber contraction speed normalized by the maximum contraction speed of muscle fiber *V*_max_. $\tilde{f_{CE}}\left(\tilde{L_{\text{MUT}}}\right)$ is the normalized active muscle force-length relationship curve and $\tilde{f_{CE}}\left(\tilde{V_{\text{MUT}}}\right)$ is the normalized active muscle force-speed relationship curve.

(6) $$\begin{array}{c} \tilde{F_{CE}}+=\frac{F_{CE}}{F_{\max}},\\ \tilde{L_{\text{MUT}}}=\frac{L_{\text{MUT}}}{L_{0}^{m}},\\ \tilde{V_{\text{MUT}}}=\frac{V_{\text{MUT}}}{V_{\max}}. \end{array}$$

The calculation method of $\tilde{f_{CE}}\left(\tilde{L_{\text{MUT}}}\right)$ and $\tilde{f_{CE}}\left(\tilde{V_{\text{MUT}}}\right)$ can be expressed as follows:

(7) $$\begin{array}{c} \tilde{f_{CE}}\left(\tilde{L_{\text{MUT}}}\right)=e^{-{\left|\tilde{L_{MUT}^{0.87}-1}/0.39\right|}^{3.19}},\\ \tilde{f_{CE}}\left(\tilde{V_{\text{MUT}}}\right)=\left\{\begin{array}{cc} \frac{1-\tilde{V_{\text{MUT}}}}{1+\tilde{V_{\text{MUT}}}}, & \tilde{V_{\text{MUT}}}\geq 0,\\ 1.8-0.8\frac{1+\tilde{V_{\text{MUT}}}}{1-30.24\tilde{V_{\text{MUT}}}}, & \tilde{V_{\text{MUT}}}<0. \end{array}\right. \end{array}$$

Passive muscle force *F*_PEE_ is produced by passive stretching of non-contractile tissue within the muscle and *F*_PEE_ is related to its own muscle fiber length *L*_MUT_, and when the muscle length exceeds the optimal muscle fiber length *L*_0_^*m*^, *F*_PEE_ can be expressed as follows:

(8) $$\begin{array}{c} F_{\text{PEE}}=F_{\max}\cdot \tilde{F_{\text{PEE}}}=F_{\max}\cdot \tilde{f_{\text{PEE}}}\left(\tilde{L_{\text{MUT}}}\right), \end{array}$$

$\tilde{F_{\text{PEE}}}$ is the normalized passive muscle force after maximum isometric *F*_max_ normalization of *F*_PEE_. $\tilde{L_{\text{MUT}}}$ is the normalized muscle fiber length after *L*_*MUT*_ normalized by the optimal muscle fiber length *L*_0_^*m*^, and $\tilde{f_{CE}}\left(\tilde{L_{\text{MUT}}}\right)$ is the normalized active muscle force-length relationship curve.

(9) $$\begin{array}{c} \tilde{f_{CE}}\left(\tilde{L_{\text{MUT}}}\right)=0.0238e^{5.31\left(∼/L_{\text{MUT}}-1\right)}. \end{array}$$

The generation of *SEE* passive tendon force *F*_*T*_ is only related to the actual length *L*_*T*_ of its own tendon at the current time.

(10) $$\begin{array}{c} F_{T}=F_{\max}\cdot \tilde{f_{\text{SEE}}}\left(\tilde{L_{T}}\right), \end{array}$$

$\tilde{f_{\text{SEE}}}\left(\tilde{L_{T}}\right)$ is the passive tendon force-length curve. $\tilde{L_{T}}$ is the normalized muscle fiber length after *L*_*T*_ normalized by the optimal tendon relaxation length *L*_*s*_^*t*^, and its normalized expression can be expressed as follows:

(11) $$\begin{array}{c} \tilde{L_{T}}=\frac{\left(L_{T}-L_{s}^{t}\right)}{L_{s}^{t}}. \end{array}$$

Muscle tissue produces muscle force by consuming metabolic energy. Tendon tissue has high energy conversion characteristics. Its energy conversion and metabolism are in balance, so it can be considered that metabolic energy is not consumed [18]. Based on the mathematical model of muscle EC of a single separated muscle, the metabolic EC of muscle fiber tissue in a gait cycle (GC) is estimated, and the specific metabolic energy power can be expressed as below.

(12) $$\begin{array}{c} P_{ME}=\alpha \cdot F_{\max}\cdot V_{\max}\cdot f_{ME}\left(\tilde{V_{\text{MUT}}}\right), \end{array}$$

$f_{ME}\left(\tilde{V_{\text{MUT}}}\right)$ is the normalized contraction speed of muscle fibers.

(13) $$\begin{array}{c} f_{ME}\left(\tilde{V_{\text{MUT}}}\right)=\left\{\begin{array}{cc} 0.23-0.16e^{-8\tilde{V_{\text{MUT}}}}, & \tilde{V_{\text{MUT}}}\geq 0,\\ 0.01-0.11\tilde{V_{\text{MUT}}}+0.06e^{23\tilde{V_{\text{MUT}}}}, & \tilde{V_{\text{MUT}}}<0. \end{array}\right.. \end{array}$$

The metabolic EC of muscle in a GC can be obtained by integrating the metabolic energy power *P*_*ME*_.

(14) $$\begin{array}{c} W_{\text{ME}}=\int P_{\text{ME}}\left(t\right)\text{dt} \end{array}$$

The article "Construction and Simulation of Biomechanical Model of Human Hip Joint Muscle-Tendon Assisted by Elastic External Tendon by Hill Muscle Model" was published in 2022. Journal: Comput Intell Neurosci.

### 2.2. Hill Muscle Optimization Model to Establish Data and Parameters

The optimized model based on the HMM was used to establish human parameters [19, 20], which were modeled with human parameters of 170 cm and 70 kg. The length of the thigh connecting rod was 434 mm; the distance of the single-joint muscle insertion point was 210 mm; the relative position of the iliopsoas pelvic attachment point was (26 mm, 22 mm, and 5 mm); the length of the moment arm at the joint was 28 mm, the physiological cross-sectional area of the muscle was 28.9 cm^2^; the muscle pinna angle was 13.9°; the relative position of the rectus femoris pelvic attachment point was (41 mm, −4 mm, and −36 mm); the length of the moment arm at the joint was 50 mm; the physiological cross-sectional area was 34.8 cm^2^; the muscle pinna angle was 12.4°; the relative position of gluteus maximus pelvic attachment points was (−88 mm, 66 mm, and −39 mm); the moment arm length at its joint was 60 mm, the physiological cross-sectional area was 46.8 cm^2^, and the muscle pinna angle was 21.0°; the moment arm length at the hamstring joint was 28 mm, the moment arm length at the lumbar joint was 28 mm, the physiological cross-sectional area was 73.0 cm^2^, and the muscle pinna angle was 11.3°.

### 2.3. Establishment of Hill Muscle Optimization Model

The movement of the human lower limb mainly occurs in the sagittal plane. The HJ MT model was constructed based on the sagittal plane. The specific results are shown in Figure 1. In order to make the model closer to the human movement mode and reduce its complexity, only the main muscles related to HJ movement were considered, including gluteus maximus, iliopsoas, rectus femoris, hamstring muscle, and passive elastic elements, of which hamstring muscle included semitendinosus, semimembranosus, and long head of biceps femoris. The mechanical properties of each muscle were represented in an HMM. The *α* of the HJ muscle was small, and considering it as 0, then the HMM simplified to the fusiform Hill model. The angle of HJ and knee joint movement was expressed by *δ* and *η*, respectively, and the angle of iliopsoas muscle and joint moment arm was *β*1, the angle of rectus femoris and joint moment arm was *β*2 and *β*3, the angle of gluteus maximus and joint moment arm was *β*4, and the angle of hamstring muscle and joint moment arm was *β*5 and *β*6.

The article "Construction and Simulation of Biomechanical Model of Human Hip Joint Muscle-Tendon Assisted by Elastic External Tendon by Hill Muscle Model" was published in 2022. Journal: Comput Intell Neurosci.

In order to make the HMM consistent with the biomechanical characteristics of the HJ when the human body is walking, the unknown parameter vector *Q*=[*H*, *I*] of the model is solved by the way of constraint optimization problem, *H* is the angle variable of the muscle force arm at the joint and the muscle force scaling variable. The calculation method is *H*=[*β*_1_, *β*_2_, *β*_3_, *β*_4_, *β*_5_, *β*_6_, *m*, *n*], and *I* is the variable of the optimal muscle fiber length of the muscle. The calculation method is *I*=[*l*_01_^*m*^, *l*_02_^*m*^, *l*_03_^*m*^, *l*_04_^*m*^]. The muscle moment calculation method of each muscle unit acting on the HJ of the optimized HMM can be expressed as follows:

(15) $$\begin{array}{c} M_{\text{MUT}}=F_{\text{MUT}}\cdot U\left(\beta \right)=F_{\max}\left(m,n\right)\cdot \tilde{F_{\text{MUT}}}\cdot U\left(\beta \right), \end{array}$$

*U*(*β*) is the vertical action arm length of each muscle force at a certain time in the GC; *m* and *n* represent the unknown scaling variable.

The calculation method of net joint moment *M*_mo_ at HJ of optimized HMM is as follows:

(16) $$\begin{array}{c} M_{\text{mo}}=M_{\text{MUT}3}+M_{\text{MUT}4}-M_{\text{MUT}1}-M_{\text{MUT}2}-M_{p}, \end{array}$$

*M*_*p*_ is the passive flexion moment generated for elastic tissue at the joint, and *M*_MUT1_ ~ *M*_MUT4_ denotes the flexion moment generated by gluteus maximus, iliopsoas, rectus femoris, and hamstring muscle, respectively.

The average difference between the model joint moment *M*_mo_ and the experimentally obtained human HJ biological moment *M*_hu_ over a GC is expressed as root mean square error (RMSE).

(17) $$\begin{array}{c} \text{RMSE}=\sqrt{\frac{\sum_{\text{i}=1}^{n}{\left(M_{\text{mo}}-M_{\text{hu}}\right)}^{2}}{n}}, \end{array}$$

*n* is the number of sampling points. Combining the constraints of each muscle parameter, the constrained optimization problem is expressed as follows:

(18) $$\begin{array}{c} \min\text{RMSE,}\\ \text{s.t}.12^{\circ }\leq \beta_{1}\leq 145^{\circ },\\ 12^{\circ }\leq \beta_{2}\leq 145^{\circ },\\ 60^{\circ }\leq \beta_{3}\leq 180^{\circ },\\ 35^{\circ }\leq \beta_{4}\leq 165^{\circ },\\ 35^{\circ }\leq \beta_{5}\leq 165^{\circ },\\ 12^{\circ }\leq \beta_{6}\leq 145^{\circ },\\ 0^{\circ }\leq \beta_{1}\leq 120^{\circ },\\ 0.5\leq m\leq 1.5,\\ 0.5\leq m\leq 1.5. \end{array}$$

The standardized passive muscles were calculated according to the known standardization $\tilde{L_{\text{MUT}}}$ combined with *PEE* kinetic equation. The standardized active muscle force $\tilde{F_{CE}}$ was obtained according to the *CE* kinetic equation, and then the actual muscle force *F*_MUT_ at a certain time of each muscle GC was calculated according to the maximum equal moment *F*_max_ of the standardized $\tilde{F_{MUT}}$ and unknown scaled variables, *U*(*β*) was calculated using the geometric relationship of the musculoskeletal system; the net joint moment of the musculoskeletal model was obtained to obtain the moment error value; the model parameters were optimized using the RMSE between the output moment of the model and the experimental moment as the solution problem, and the optimal solution of *H* was obtained using MATLAB genetic algorithm.

The article "Construction and Simulation of Biomechanical Model of Human Hip Joint Muscle-Tendon Assisted by Elastic External Tendon by Hill Muscle Model" was published in 2022. Journal: Comput Intell Neurosci.

The subset *I* constrained optimization problem for the unknown vector *Q* can be expressed as follows:

(19) $$\begin{array}{c} \min b_{\min},\\ \text{s.t}.\;0\leq b\left(t\right)\leq 1, \end{array}$$

*b*_min_ denotes the minimum value of muscle activation during one GC.

The optimal variables *m* and *n* are substituted into the dynamic equation of model muscle to solve *F*_MUT_, the normalized muscle fiber length $\tilde{L_{T}}$, and actual contraction speed *V*_MUT_ under the corresponding tendon force are calculated according to the force-length dynamic equation of the tendon, and at the same time *L*_MUT_ is substituted into the *PEE* dynamic equation to solve *F*_PEE_ and *F*_*CE*_. The muscle activation *b* is obtained by introducing them into the *CE* dynamic equation according to the obtained parameters, and finally the optimal solution of *I* is obtained according to the constrained optimization problem. The specific flow for solving the scaling variable *H* and the optimal fiber length variable *I* is given in Figure 2.

EET can provide auxiliary flexion moment for HJ during lower limb walking, and based on its effect, the external elastic tendon is assumed to be a passive linear torsional spring parallel to the HJ. For an EET with a stiffness of *J*, its resulting flexion moment *M*_J_ during walking of the lower limb can be expressed as follows:

(20) $$\begin{array}{c} M_{\text{J}}\left(t\right)=\left\{\begin{array}{cc} 0, & \delta \geq 0,\\ J\cdot \delta \left(t\right), & \delta <0. \end{array}\right. \end{array}$$

EET acts directly with human HJ flexor muscle group [21]. During the auxiliary period of EET, the calculation method of residual total flexion biological moment *M*_Re_ provided by rectus femoris and iliopsoas muscle based on Hill muscle optimization model can be expressed as follows:

(21) MRe=MI+MR−MJ,MJ<MT,

*M*_*I*_ represents the moment of iliopsoas muscle; *M*_*R*_ represents the moment of rectus femoris; *M*_*T*_ represents *M*_*J*_ less than the total flexion moment of flexor at HJ during natural walking.

The article "Construction and Simulation of Biomechanical Model of Human Hip Joint Muscle-Tendon Assisted by Elastic External Tendon by Hill Muscle Model" was published in 2022. Journal: Comput Intell Neurosci.

The additional calculation method of resistance moment provided by gluteus maximus and hamstring muscle based on Hill muscle optimization model is as follows:

(22) $$\begin{array}{c} M_{\text{Ex}}=M_{I}+M_{R}-M_{J},M_{J}>M_{T}. \end{array}$$

The biological moment solution and biomechanical simulation framework of each muscle of the model under the action of EET are shown in Figure 3.

### 2.4. Simulation Test Conditions of HJ MT Biomechanical Model

The simulation experiment of HJ muscle tendon biomechanical model was mainly carried out in the software of automatic dynamic analysis of mechanical systems (ADAMS). It mainly provided constraint base and force base centered on the user through ADAMS/View module, and gathers the functions of interactive image, simulation calculation, and result analysis together to effectively carry out modeling and simulation. Moreover, MATLAB program was used for programming. The program was mainly composed of data input, data calculation and solution, data output, and graphical interface.

## 3. Results

### 3.1. Evaluation of Optimized HMM Performance

Firstly, the biomechanical properties of human lower limb walking under the optimized HMM were evaluated from the joint level. During a GC, the change trends of the output joint moment of the optimized HMM and the biological moment of the human HJ were basically the same, showing a trend of first increase and then decrease. The similarity of the output joint moment of the optimized HMM and the biological moment curve of the human HJ was compared using the coefficient *r*^2^ and RMSE. The results showed that the HJ moment *r*^2^ = 0.883, RMSE = 0.18 Nm/kg (Figure 4(a)). The total metabolic EC power during one GC of the HJ under the optimized HMM was statistically analyzed using the muscle energetics equation, and it was in a fluctuating state during one GC, with an average metabolic EC of (243.77 ± 1.59) *J* (Figure 4(b)).

The validity of the optimized HMM was further evaluated from the muscle level, and the results showed that the muscle activation curves of gluteus maximus, iliopsoas, rectus femoris, and hamstring muscle under the optimized HMM tended to be similar to the test activation curve during one GC; *r*^2^ = 0.875, RMSE = 0.19 Nm/kg for iliopsoas; *r*^2^ = 0.890, RMSE = 0.15 Nm/kg for rectus femoris; *r*^2^ = 0.892, RMSE = 0.16 Nm/kg for gluteus maximus; and *r*^2^ = 0.879, RMSE = 0.18 Nm/kg for hamstring muscle (Figure 5).

The article "Construction and Simulation of Biomechanical Model of Human Hip Joint Muscle-Tendon Assisted by Elastic External Tendon by Hill Muscle Model" was published in 2022. Journal: Comput Intell Neurosci.

### 3.2. Analysis of Moment Change of Human HJ under Different EET Stiffness

The changes of human auxiliary moment and human HJ biomechanical moment under different EET stiffness were analyzed. With the increase of EET stiffness during GC, the corresponding auxiliary moment showed a significant trend of first reduction and then increase, and finally tended to be stable. In the range of 35%∼65% of GC, the auxiliary moment showed a significant downward trend with the increase of EET stiffness. When the EET stiffness was 0 Nm/rad, the auxiliary flexion moment showed a stable state (Figure 6(a)). With the increase of EET stiffness, in the range of 35%∼65% of GC, when the EET stiffness of human body was less than 200 Nm/rad, the biological moment of human HJ gradually decreased with the increase of EET stiffness, and when the EET stiffness of human body was greater than 200 Nm/rad, the biological moment of human HJ gradually increased with the increase of EET stiffness (Figure 6(b)).

By analyzing the changes of the total flexor moment of the HJ under different EET stiffness (Figure 7(a)), the total flexor moment of the HJ increased significantly with the increase of the EET stiffness in the range of 35% ∼ 65% of the GC. When the EET stiffness was less than 200 Nm/rad, the total flexor moment of the HJ decreased first and then increased with the decrease of the EET stiffness (Figure 7(a)). With the increase of EET stiffness, the total moment of human HJ extensor increased significantly in the range of 35%∼65% of GC. When the EET stiffness was greater than 200 Nm/rad, the increase range of total moment of extensor increased significantly (Figure 7(b)).

### 3.3. Analysis on the Change of Muscle Moment Distribution Coefficient (MDC) under Different EET Stiffness

The change of muscle MDC under different EET stiffness was analyzed. With the increase of EET stiffness, the change trend of MDC of different muscles was significantly different. When the stiffness of the external tendon was less than 200 Nm/rad, the MDC of iliopsoas muscle gradually decreased with the increase of the stiffness of the external tendon. When the stiffness of the external tendon was greater than 350 Nm/rad, the MDC of iliopsoas muscle gradually tended to a stable state with the increase of the stiffness of the external tendon (Figure 8(a)). When the stiffness of the external tendon was less than 250 Nm/rad, the rectus femoris MDC gradually increased with the increase of the stiffness of the external tendon. When the stiffness of the external tendon was greater than 250 Nm/rad, the rectus femoris MDC gradually decreased to zero with the increase of the stiffness of the external tendon (Figure 8(b)). With the increase of external tendon stiffness (ETS), gluteus maximus MDC gradually increased (Figure 8(c)). With the increase of ETS, hamstring muscle MDC showed a gradual downward trend (Figure 8(d)).

The article "Construction and Simulation of Biomechanical Model of Human Hip Joint Muscle-Tendon Assisted by Elastic External Tendon by Hill Muscle Model" was published in 2022. Journal: Comput Intell Neurosci.

### 3.4. Analysis of Muscle Moment Changes under Different EET Stiffness

The moment changes of different muscles under different EET stiffness were analyzed. With the increase of EET stiffness, the moment changes of different muscles were obviously different. In the range of 35% ∼ 65% of GC, with the increase of ETS, the moment of iliopsoas and rectus femoris muscle gradually decreased. When the ETS was greater than 600 Nm/rad, the moment of iliopsoas and rectus femoris gradually approached zero (Figures 9(a) and 9(b)). In the range of 35% ∼ 65% of GC, the muscle moment of gluteus maximus and hamstring muscle gradually increased with the increase of ETS (Figures 9(c) and 9(d)).

### 3.5. Analysis of Muscle Force Change under Different EET Stiffness

The force changes of each muscle under different EET stiffness were analyzed, and the moment changes of different muscles were significantly different with the increase of EET stiffness. In the range of 35% ∼ 65% of GC, the iliopsoas muscle force gradually decreased with the increase of ETS (Figure 10(a)); in the range of 15% ∼ 65% of GC, the rectus femoris muscle force gradually decreased with the increase of ETS (Figure 10(b)); and in the range of 35% ∼ 60% of GC, the gluteus maximus and hamstring muscle forces gradually increased with the increase of ETS (Figures 10(c) and 10(d)).

### 3.6. Analysis of Muscle Power Changes under Different EET Stiffness

The change of muscle power under different EET stiffness was analyzed. With the increase of EET stiffness, the change trend of different muscle power was clearly different. In a GC, the muscle power of iliopsoas muscle decreased first and then increased. In the range of 55% ∼ 65% of the GC, with the increase of ETS, the muscle power of iliopsoas muscle gradually increased (Figure 11(a)); in one GC, the muscle power of rectus femoris decreased first and then increased. In the range of 60% ∼ 85% of GC, the muscle power of rectus femoris gradually decreased and tended to zero with the increase of ETS (Figure 11(b)). In the range of 35% ∼ 65% of GC, the muscle power of gluteus maximus gradually increased with the increase of ETS (Figure 11(c)). In the range of 35% ∼ 65% of GC, with the increase of ETS, hamstring muscle power gradually increased. When the ETS was 0, hamstring muscle power was zero (Figure 11(d)).

The changes of muscle mechanical work under different ETS were analyzed. With the increase of EET stiffness, the mechanical work of HJ decreased gradually. When the EET stiffness was less than 200 Nm/rad, the mechanical work of muscle unit showed a downward trend, and when the EET stiffness was greater than 200 Nm/rad, the mechanical work of muscle unit and muscle fiber showed an upward trend. With the increase of EET stiffness, the mechanical work of tendon did not change. With the increase of EET stiffness, the mechanical work of knee joint gradually decreased (Figure 12).

The article "Construction and Simulation of Biomechanical Model of Human Hip Joint Muscle-Tendon Assisted by Elastic External Tendon by Hill Muscle Model" was published in 2022. Journal: Comput Intell Neurosci.

## 4. Discussion

The results showed that the changing trends of the output joint moment of the optimized HMM and the biological moment of the human HJ were basically the same, showing a trend of first increase and then decrease, with the HJ moment *r*^2^ = 0.883 and RMSE = 0.18 Nm/kg. For the general musculoskeletal model, when the moment curve *r*^2^ was greater than 0.883 and the RMSE value was less than 0.2 Nm/kg, it could be considered that the moment curve fitting had a higher goodness, and the established model was close to the mechanical characteristics of the human musculoskeletal [22]. Optimized HMM can effectively reproduce the biological characteristics of human HJ at joint moment level. The characteristics of the established model were further evaluated from the muscle level, and the results showed that the muscle activation curves of gluteus maximus, iliopsoas, rectus femoris, and hamstring muscles under the optimized HMM had similar trends to the test activation curves, and the shape of the activation curves of different muscle tests was similar to the results of Bogey and Barnes (2017) [23]. The total metabolic energy consumption power curve of the model muscle in a gait cycle was calculated by muscle energy equation. The result revealed the average metabolic EC of the HJ was (243.77 ± 1.59) J. It has been pointed out that the total metabolic EC rate produced during normal walking in the human body was (5.20 ± 0.91) W/kg [24], the net metabolic EC rate was about (3.39 ± 0.58) W/kg [25], and the net metabolic rate was (1.81 ± 0.33) W/kg [26]. During walking in the human body, the energy consumed by the HJ muscle accounted for 9/20 of the total metabolic energy. Therefore, the total metabolic EC rate of walking in the human body based on the optimized HMM was 6.22 W/kg, which was consistent with the metabolic EC level of the HJ muscle found in the current relevant studies [27, 28]. In conclusion, the optimized HMM can effectively reproduce the biological characteristics of human HJ at joint moment level, joint level, and muscle level.

With the increase of EET stiffness in GC, the corresponding auxiliary moment showed a significant trend of first reduction and then increased and finally tended to be stable, and in the range of 35% ∼ 65% of GC the auxiliary moment showed a significant downward trend with the increase of EET stiffness. When the EET stiffness of the human body was less than 200 Nm/rad, the biological moment of the human HJ gradually decreased with the increase of the EET stiffness, and when the EET stiffness of the human body was greater than 200 Nm/rad, the biological moment of the human HJ gradually increased with the increase of the EET stiffness, and the total moment of the extensor muscle increased significantly. There was a significant antagonistic effect among human flexor and extensor muscle groups [29], and the flexion moment generated by the HJ flexor muscles was obviously greater than the joint moment during human walking [30]. When the elastic external stiffness increased to 200 Nm/rad, the HJ moment value was significantly smaller than the auxiliary flexion moment value but the HJ extensor moment did not change during the reduction of the flexor moment. When the EET stiffness was greater than 200 Nm/rad, the human HJ flexor muscles can only provide energy through the EET auxiliary interval, which in turn leaded to a decrease in the flexion moment [31], and as the EET stiffness gradually became larger, the HJ moment gradually changed from the flexion moment to the extension moment [32]. In the range of 35% ∼ 65% of GC, the moment of iliopsoas and rectus femoris muscles gradually decreased with the increase of ETS, and the moment of iliopsoas and rectus femoris muscles gradually approached to zero when the ETS was greater than 600 Nm/rad. With the auxiliary of EET, the degree of auxiliary of the iliopsoas was more significant, and gluteus maximus appeared as a resistant muscle when the force generated by EET stiffness gradually increased. This was because monoarticular muscles such as iliopsoas and gluteus maximus were mainly driving joint movements [33], while biarticular muscles such as rectus femoris and hamstring muscle were mainly responsible for energy transfer between joints [34]. With the auxiliary of EET, the human control system tended to be more stable control than motor control [35]. In order to maintain the stability of the human motor system, single-joint muscles play an important role in it [36]. Therefore, the biomechanical parameters of iliopsoas and gluteus maximus changed most significantly with the auxiliary of EET. In the range of 35% ∼ 65% of GC, with the increase of ETS, the iliopsoas muscle force gradually increased, the rectus femoris muscle force gradually decreased, and the gluteus maximus and hamstring muscle forces gradually increased. The force of both iliopsoas and rectus femoris muscles decreased as the stiffness of EET auxiliary increased, and their corresponding muscle fiber lengths showed an increasing trend. The compliance of the tendon can have a significant effect on the length of the muscle fibers [37], and the tendon compliance of the iliopsoas muscle was small and short in length, so its muscle fiber length increased less; the tendon compliance of rectus femoris was long and flexible, but its muscle force decreased less, which in turn leaded to a smaller increase in its muscle fiber length.

The article "Construction and Simulation of Biomechanical Model of Human Hip Joint Muscle-Tendon Assisted by Elastic External Tendon by Hill Muscle Model" was published in 2022. Journal: Comput Intell Neurosci.

## 5. Conclusion

A biomechanical model of human HJ MT assisted by EET was established based on the HMM, and it was found by simulation experiment that muscle activation had a significant effect on HJ muscle moment, muscle force as well as mechanical work changes with EET assistance, and metabolic EC during human walking could be reduced with EET assistance. However, there are still some shortcomings, only the biomechanical changes of human HJ MT assisted by EET are preliminarily explored and they are not compared with the ankle joint. In the future, the biomechanical properties of the two will be further compared. The optimized HMM can reflect the law of human motion, and complete the simulation test of typical movements of HJ, which provides a new idea for the analysis of energy migration of lower limb musculoskeletal system.

## Figures and Tables

**Figure 1:** Musculoskeletal model of HJ. (a) Main muscles and elements related to movement of HJ musculoskeletal model; (b) parameters related to HJ musculoskeletal model.

**Figure 2:** The specific flow chart for solving the shrinkage variable H and the optimal fiber length variable (I) construction of Biomechanical Model of HJ MT assisted by EET.

**Figure 3:** Biological moment solution and biomechanical simulation framework of each muscle.

**Figure 4:** Power change curve of HJ moment and total metabolic EC under optimized HMM. (a) HJ moment compared with human biological moment; (b) total metabolic (EC power).

**Figure 5:** Change curve of different muscle activation data under optimized HMM. (a) Iliopsoas; (b) rectus femoris; (c) gluteus maximus; (d) hamstring muscle.

**Figure 6:** Changes of auxiliary moment and HJ biomechanical moment under different EET auxiliary stiffness. (a) Change curve of human auxiliary moment under the same EET stiffness; (b) change curve of human HJ biological moment under the same EET stiffness.

**Figure 7:** Moment change curve under different EET auxiliary stiffness. (a) Total flexor moment; (b) total extensor moment.

**Figure 8:** Change curve of muscle MDC under different EET stiffness.

**Figure 9:** Muscle moment change curve under different EET auxiliary stiffness.

The article "Construction and Simulation of Biomechanical Model of Human Hip Joint Muscle-Tendon Assisted by Elastic External Tendon by Hill Muscle Model" was published in 2022. Journal: Comput Intell Neurosci.

**Figure 10:** Muscle force change curve under different EET stiffness.

**Figure 11:** Muscle power change curve under different EET stiffness.

**Figure 12:** Muscle mechanical work change curve under different ETS.

## Data Availability

The datasets used during the current study are available from the corresponding author on reasonable request.

## References

[1] Mendonça L. D., Ocarino J. M., Bittencourt N. F. N., Macedo L. G., Fonseca S. T. (2018). Association of hip and foot factors with patellar tendinopathy (Jumper’s Knee) in Athletes. *Journal of Orthopaedic & Sports Physical Therapy*.

[2] Kainz H., Schwartz M. H. (2021). The importance of a consistent workflow to estimate muscle-tendon lengths based on joint angles from the conventional gait model. *Gait & Posture*.

[3] Audenaert E. A., Khanduja V., Bauwens C., Van Hoof T., Pattyn C., Steenackers G. (2019). A discrete element model to predict anatomy of the psoas muscle and path of the tendon: Design implications for total hip arthroplasty. *Clinical Biomechanics*.

[4] Chen W., Wu S., Zhou T., Xiong C. (2018). On the biological mechanics and energetics of the hip joint muscle-tendon system assisted by passive hip exoskeleton. *Bioinspiration & Biomimetics*.

[5] Chicoine D., Bouchard M., Laurendeau S., Moisan G., Belzile E. L., Corbeil P. (2021). Biomechanical effects of three types of foot orthoses in individuals with posterior tibial tendon dysfunction. *Gait & Posture*.

[6] Wade L., Lichtwark G. A., Farris D. J. (1985). Joint and muscle-tendon coordination strategies during submaximal jumping. *Journal of Applied Physiology*.

[7] Martín-Sosa E., Martínez-Reina J., Mayo J., Ojeda J. (2019). Influence of musculotendon geometry variability in muscle forces and hip bone-on-bone forces during walking. *PLoS One*.

[8] Burzyński S., Sabik A., Witkowski W., Łuczkiewicz P. (2021). Influence of the femoral offset on the muscles passive resistance in total hip arthroplasty. *PLoS One*.

[9] Hapa O., Demirkıran N. D., Hüsemoğlu B., Edizer M., Havitçioğlu H. (2018). Anatomic implications of lesser trochanterplasty. *Acta Orthopaedica et Traumatologica Turcica*.

[10] Cerda-Lugo A., González A., Cardenas A., Piovesan D. (2020). Modeling the neuro-mechanics of human balance when recovering from a fall: a continuous-time approach. *BioMedical Engineering Online*.

[11] Tan Y., Fu Z., Duan L. (2021). Hill-based musculoskeletal model for a fracture reduction robot. *International Journal of Medical Robotics and Computer Assisted Surgery*.

[12] Siebert T., Stutzig N., Rode C. (2018). A hill-type muscle model expansion accounting for effects of varying transverse muscle load. *Journal of Biomechanics*.

The article "Construction and Simulation of Biomechanical Model of Human Hip Joint Muscle-Tendon Assisted by Elastic External Tendon by Hill Muscle Model" was published in 2022. Journal: Comput Intell Neurosci.

[13] Rockenfeller R., Günther M., Stutzig N. (2020). Exhaustion of Skeletal Muscle Fibers Within Seconds: Incorporating Phosphate Kinetics Into a Hill-Type Model. *Frontiers in Physiology*.

[14] Xiong B., Zeng N., Li Y. (2020). Determining the Online Measurable Input Variables in Human Joint Moment Intelligent Prediction Based on the Hill Muscle Model. *Sensors*.

[15] Bujalski P., Martins J., Stirling L. (2018). A Monte Carlo analysis of muscle force estimation sensitivity to muscle-tendon properties using a Hill-based muscle model. *Journal of Biomechanics*.

[16] Heinen F., Sørensen S. R., King M. (2019). Muscle-Tendon Unit Parameter Estimation of a Hill-Type Musculoskeletal Model Based on Experimentally Obtained Subject-Specific Torque Profiles. *Journal of Biomechanical Engineering*.

[17] Palladino J. L. Functional Requirements of a Mathematical Model of Muscle Contraction.

[18] Guo J., Sun Y., Hao Y., Cui L., Ren G. (2020). A mass-flowing muscle model with shape restrictive soft tissues: correlation with sonoelastography. *Biomechanics and Modeling in Mechanobiology*.

[19] Kleinbach C., Martynenko O., Promies J., Haeufle D. F. B., Fehr J., Schmitt S. (2017). Implementation and validation of the extended Hill-type muscle model with robust routing capabilities in LS-DYNA for active human body models. *BioMedical Engineering Online*.

[20] Shao Z., Wu Q., Chen B., Wu H. (2019). Force and deformation transmission characteristics of a compliant tendon-sheath actuation system based on Hill-type muscle model. *Proceedings of the Institution of Mechanical Engineers - Part H: Journal of Engineering in Medicine*.

[21] Rockenfeller R., Günther M. (2017). Hill equation and Hatze’s muscle activation dynamics complement each other: enhanced pharmacological and physiological interpretability of modelled activity-pCa curves. *Journal of Theoretical Biology*.

[22] Mohammadi Nejad Rashty A., Grimmer M., Seyfarth A. (2021). Hopping frequency influences elastic energy reuse with joint series elastic actuators. *Journal of Biomechanics*.

[23] Bogey R. A., Barnes L. A. (2017). Estimates of individual muscle power production in normal adult walking. *Journal of NeuroEngineering and Rehabilitation*.

[24] Martin J. C., Nichols J. A. (2018). Simulated work-loops predict maximal human cycling power. *Journal of Experimental Biology*.

[25] Lim Y. P., Lin Y. C., Pandy M. G. (2017). Effects of step length and step frequency on lower-limb muscle function in human gait. *Journal of Biomechanics*.

[26] Zumbrunn T., Patel R., Duffy M. P. (2018). Cadaver-Specific Models for Finite-Element Analysis of Iliopsoas Impingement in Dual-Mobility Hip Implants. *The Journal of Arthroplasty*.

The article "Construction and Simulation of Biomechanical Model of Human Hip Joint Muscle-Tendon Assisted by Elastic External Tendon by Hill Muscle Model" was published in 2022. Journal: Comput Intell Neurosci.

[27] Allen V. R., Kambic R. E., Gatesy S. M., Hutchinson J. R. (2017). Gearing effects of the patella (knee extensor muscle sesamoid) of the helmeted guineafowl during terrestrial locomotion. *Journal of Zoology*.

[28] Zhu M., Musson D., Oliver M., Firth E., Cornish J., Munro J. (2022). Modelling gluteus medius tendon degeneration and repair in a large animal model. *Archives of Orthopaedic and Trauma Surgery*.

[29] Sedlmayr J. C., Bates K. T., Wisco J. J., Schachner E. R. (2022). Revision of hip flexor anatomy and function in modern humans, and implications for the evolution of hominin bipedalism. *The Anatomical Record*.

[30] Souza T. R., Schallig W., Veerkamp K. (2022). Muscle actions on crossed and non-crossed joints during upright standing and gait: A comprehensive description based on induced acceleration analysis. *Journal of Biomechanics*.

[31] Tsai L. C., Ko Y. A., Hammond K. E., Xerogeanes J. W., Warren G. L., Powers C. M. (2017). Increasing hip and knee flexion during a drop-jump task reduces tibiofemoral shear and compressive forces: implications for ACL injury prevention training. *Journal of Sports Sciences*.

[32] Dick T. J. M., Punith L. K., Sawicki G. S. (2019). Humans falling in holes: adaptations in lower-limb joint mechanics in response to a rapid change in substrate height during human hopping. *Journal of The Royal Society Interface*.

[33] Dick T. J. M., Clemente C. J., Punith L. K., Sawicki G. S. (2021). Series elasticity facilitates safe plantar flexor muscle-tendon shock absorption during perturbed human hopping. *Proceedings of the Royal Society B: Biological Sciences*.

[34] Nuckols R. W., Takahashi K. Z., Farris D. J., Mizrachi S., Riemer R., Sawicki G. S. (2020). Mechanics of walking and running up and downhill: A joint-level perspective to guide design of lower-limb exoskeletons. *PLoS One*.

[35] Tokur D., Grimmer M., Seyfarth A. (2020). Review of balance recovery in response to external perturbations during daily activities. *Human Movement Science*.

[36] Miller S. E., Segal A. D., Klute G. K., Neptune R. R. (2018). Hip recovery strategy used by below-knee amputees following mediolateral foot perturbations. *Journal of Biomechanics*.

[37] Shell C. E., Segal A. D., Klute G. K., Neptune R. R. (2017). The effects of prosthetic foot stiffness on transtibial amputee walking mechanics and balance control during turning. *Clinical Biomechanics*.

